# Public School Adolescents Had Increased Odds of Being Willing to Uptake HPV Vaccinations Owing to Sociodemographic and Healthcare Access Features in Bahir Dar City, Ethiopia

**DOI:** 10.1155/2023/2663815

**Published:** 2023-04-12

**Authors:** Birhanu Feleke Shitu, Desta Debalkie Atnafu, Yeshambel Agumas

**Affiliations:** ^1^Department of Public Health, Addis Continental Institute of Public Health, Bahir Dar, Ethiopia; ^2^Department of Health Systems Management and Health Economics, School of Public Health, College of Medicine and Health Science, Bahir Dar University, Bahir Dar, Ethiopia; ^3^International Centre for Evidence in Disability, London School of Hygiene & Tropical Medicine, London WC1E 7HT, UK

## Abstract

**Background:**

Cervical cancer is one of the most prevalent and fatal malignancies in women worldwide. Despite the fact that vaccination is an effective method in reducing cervical cancer, its uptake varies between public and private school adolescents and remains a challenge in low- and middle-income countries, including Ethiopia. Empirical evidence on how much variation there is among public and private school adolescent in their willingness to uptake human papillomavirus (HPV) vaccination is also limited. Thus, the aim of this study was to compare levels of willingness to uptake HPV vaccination among public and private school female adolescents and associated factors in Bahir Dar City, Ethiopia.

**Methods:**

A comparative cross-sectional study was conducted on 844 adolescents aged 10 to 19 in primary schools in Bahir Dar, Ethiopia. Multistage sampling was used. A self-administered, structured, and pretested questionnaire was used to collect data. The determinants of willingness to accept HPV vaccination were identified using logistic regression, and exploratory factor analyses were performed to determine load and mean. The level of statistical significance was determined using a *P* - value of 0.05.

**Results:**

The overall proportion of willing to uptake HPV vaccination was 50.6% (95% CI: 47.4-54), whereas in public and private primary schools, the magnitude was 61% (95% CI: 56.3-65.4%) and 40.2% (95% CI: 35.6-44.9), respectively. In terms of willingness to uptake HPV vaccination, the odds were likely to be significantly higher among those whose mothers had a postsecondary education (AOR = 2.0, 95% CI: 1.29-3.05), a high cue to action (AOR = 1.92, 95% CI: 1.20-3.05), and high self-efficacy (AOR = 2.34, 95% CI: 1.58-3.48). High perceived barriers likely decreased the willingness to uptake HPV vaccination (AOR = 0.49, 95% CI: 0.34-0.70).

**Conclusion:**

Adolescent girls in public primary schools were more likely to uptake HPV vaccination than those in private provided that income status and socioeconomic factors became less important. Willingness to uptake HPV vaccination was found to be low as compared to the WHO target for Ethiopian context and was influenced by maternal education status, perceived barriers, cues to action, and self-efficacy. As a result, greater emphasis should be placed on implementing a school-based and maternal educational program on cervical cancer prevention and control focusing on the behavioral contexts.

## 1. Background

The human papillomavirus (HPV) is the virulence responsible for the most common oncogenic cervical infection in the world. It has been linked to cancers of the larynx, oropharynx, vulvar, cervix, anus, and vagina [1, 2]. Globally, cervical cancer is the fourth most common cancer in women in 2020, with 604000 new cases and 342000 deaths. The majority of new cases and fatalities, approximately 90%, occurred in low- and middle-income countries [3]. Ethiopia has a high prevalence of cervical cancer, with variations from region to region [4]. Unless measures are taken to control and reduce the health burden of cervical cancer among adolescents, the prevalence of HPV among young women under the age of 25 has risen to the highest level in the world [5].

HPV is the most common cause of infections contracted through sexual contact. HPV was found in 99.7% of all cervical cancer cases diagnosed in the 1990s, and ongoing high-risk HPV infection contributes to cervical cancer development [6, 7]. HPVs 16 and 18 are responsible for approximately 70% of all invasive cervical cancer cases worldwide [8]. The use of vaccines, on the other hand, is effective in disease prevention. Gardasil, the first HPV vaccine, was approved by the US Food and Drug Administration (FDA) in June 2006 [9]. It is a quadrivalent vaccine that protects against HPV types 16 and 18, as well as HPV 6 and HPV 11, which are thought to cause at least 80% of genital warts [10]. Cervarix, a bivalent HPV vaccine, was also approved in 2009. HPV vaccination is in general the most effective method of preventing cervical cancer by reducing the frequency of HPV infection, particularly in developing countries and regions where population-based comprehensive national cervical cancer screenings are not feasible [11–13].

Prepuberty girls aged 9-14 years are the primary target group for HPV vaccination, according to the World Health Organization (WHO) [14]. The WHO recommends that middle school–aged girls to be the primary target populations for HPV vaccination in Ethiopia. Despite these recommendations, maintaining high HPV vaccine uptake among eligible adolescents is difficult. Surprisingly, according to a WHO report, 16 million adolescents who had their first sexual experience became pregnant unintentionally [15]. Early sexual activity raises the risk of HPV, HIV, and other STIs in adolescents [16, 17]. Up to 25% of adolescents in sub-Saharan Africa have made a sexual debut before the age of 15 [18]. In Ethiopia, however, 62% of women have their first sexual experience before the age of 18, and 58% marry before the age of 18, increasing the risk of an early sexual debut followed by cervical infection [19].

Several countries have conducted studies on the attitudes of physician, parents, and teenagers toward knowledge of HPV infection and HPV vaccination and the fact that the uptake of the HPV vaccine is dependent on a number of factors, including sociodemographics, awareness of and knowledge about HPV infection, type of school enrolment, and adolescents' perception toward HPV vaccination [20, 21].

As far as our knowledge is concerned, little is known about the knowledge of parents toward HPV vaccination and HPV vaccine uptake and associated factors, and school students were the potential with bad attitude toward HPV vaccination uptake [22–24]. Since the HPV vaccine was only recently introduced in Ethiopia, more research is therefore needed to determine the adolescents' willingness to uptake HPV vaccine. The actual difference in willingness to uptake HPV vaccine among adolescents attending public versus privately owned schools in Ethiopia has yet to be determined, and the findings of this study could provide policy insight into how to improve vaccination coverage and utilization. It is critical to develop policies governing how HPV vaccination should be given priority in the cervical cancer control program. Thus, the aim of this study was to compare the willingness to uptake HPV vaccination between public and private junior middle school students in Bahir Dar City, Ethiopia, and to identify the factors associated with willingness of HPV vaccination uptake.

## 2. Methods

### 2.1. Study Setting and Participants

Bahir Dar City is the capital city of the Amhara National Regional State. It is located 565 kilometers from Addis Ababa, the capital city of Ethiopia. According to the Bahir Dar City administrative plan commission and the city health sector information office, approximately 21% of adolescents aged 10 to 19 years old are living in Bahir Dar. With a total of 35,598 students, the city has 64 elementary schools, 38 of which are public-owned and the 26 are private. Six thousand six hundred students attended private schools, while 28,933 attended public-run primary schools [25]. All female adolescent girls aged 10-19 years in the selected primary schools in Bahir Dar City administration were included in the study. Adolescent girls aged 10 to 19 years who had a history of vaccine-related adverse events and were absent during the data collection period were excluded from the study.

#### 2.1.1. Study Design and Period

A comparative cross-sectional study design was applied from September 1 to October 30, 2021, to collect data on female adolescents enrolled in primary schools, Bahir Dar City administration.

### 2.2. Sample Size Estimation and Sampling Method

The sample size was calculated using single proportion formula in Epi Info software version 7. The study was designed with a 5% margin of error, 95% confidence interval, 10% nonresponse rate, ratio of 1 : 1 for private versus public schools, and a design effect of 2. Since the school adolescent females' willingness to uptake HPV vaccination was unknown, we took 50% assumption for willingness to uptake HPV vaccination, and thus, the estimated final sample size was 844 (422 students from the private and 422 students from the public primary schools). The sample size was determined for each variable. However, the exposure variable with the largest sample size was chosen. To recruit study participants, multistage sampling followed by stratified and simple random sampling method was used. Approximately 13 schools were chosen at random from a pool of 64. Only eight and five schools were taken from school items in proportion to a number of the schools in public versus private, respectively. The calculated sample size was assigned to those primary schools using a probability proportional to size method, with the number of adolescent female students used as a measure of size. Simple random sampling was used to select the required number of adolescent female students in each section of the selected primary schools.

### 2.3. Operational Definition

Willingness to use HPV vaccination by adolescents was measured using the question “are you willing to vaccinate for HPV vaccination against HPV infection?” with responses either Yes or No. A 14-point knowledge score questions was used to assess knowledge of HPV vaccination among school adolescents. Each correct response received a score of one, while incorrect responses received a score of zero. Adolescents with overall scores of 75% or greater were considered to have “good knowledge,” while those with scores lower than 75% were considered to have “poor knowledge.”

### 2.4. Data Collection Tools and Methods

To collect data, a structured, pretested, and self-administered questionnaire was used. Before the first day of data collection, families or guardians were sent informed consent forms to sign. All the participants held self-administered interviews outside of the classroom at school to guarantee that they were answered freely and honestly. Four female BSc nurses, who collected data, were supervised by two female MPH/RH specialists. The data were collected on sociodemographic variables (age, school grade, religion, maternal education status, maternal occupation, and family marital status) and knowledge-related characteristics (information about cervical cancer, information about HPV, cervical cancer is caused by HPV, and information about the HPV vaccine). HPV vaccination and healthcare access–related characteristics were also considered. The health belief model constructs (perceived susceptibility, perceived severity, perceived benefit, perceived barrier, cue to action, and self-efficacy) were used to assess adolescents' behavior toward HPV vaccination and its uptake. The constructs of health belief theoretical behavioral model were measured using a five-point Likert scale questions (strongly disagree, disagree, neither agree nor disagree, agree, and strongly agree). A 4-item scale and a 12-item scale were employed in the first segment to evaluate HPV severity and susceptibility, respectively. The perceived benefit of HPV vaccination was evaluated using a 5-item scale, and the perceived barriers to HPV vaccination were evaluated using an 11-item scale. The final scales consisted of a self-efficacy measure with 12 items and cues to action for HPV vaccination uptake with 9-item scale. The perceived susceptibility, severity, benefits, barriers, cues to action, and self-efficacy measures were all found to be reliable by the item-total correlation reliability test, with a correlation *r* calculated of ≥0.20 and a Cronbach alpha of 0.87 indicating that all items were reliable. Finally, using the principal component analysis of the rotated factor analysis, the explanation of each construct and the overall were summarized so that the actual influence of each construct and overall, toward willing to accept human papillomavirus vaccination, was determined.

### 2.5. Data Analysis and Management

Data were coded and entered into EpiData version 3.5.1 statistical software before being exported to SPSS for further analysis. The adolescent female students were described using frequencies and proportions in relation to the variables studied. Tables were used to present the data. To compare willingness to uptake HPV vaccination between public and private primary schools, the *X*^2^ test was used. Using bivariable binary logistic regression, variables with a *P* value of 0.25 were considered and fitted for final model, i.e., multivariable logistic regression analysis, to identify the independent determinants of willingness to uptake HPV vaccination. The strength of association was determined using adjusted odds ratios with 95% confidence intervals. The Hosmer-Lemeshow goodness-of-fit test showed that the model was fitted to the data (*P* value = 0.163).

### 2.6. Ethical Consideration

The institutional review board of Bahir Dar University granted an ethical clearance letter (IRB 3016/2021). The Amhara Health Institute provided the permission support letter to the Bahir Dar City Health Department, and the letter of support was also delivered to each primary schools. Following that, the school director granted permission to the class representatives. After the informed consent forms were sent to sign, written informed consents were obtained from all families or guardians of the primary school students. Daughters whose families/guardians refused for signing were provided full autonomy not to participate in the study.

## 3. Results

A total of 820 adolescent girls participated in the study with a response rate of 97.1%.

### 3.1. Sociodemographic Characteristics

The mean age of adolescent girls between public (13.86 (1.76)) and private (13.76(1.754)) primary schools was nearly the same in magnitude; however, there was a significant difference in age group between public and private primary school students. The variables maternal education, parental marital status, religion, student grade level, and maternal occupation, on the other hand, did not show any variation between public and private primary school students. When compared to private primary school students, nearly half of the mothers whose daughters were enrolled in public primary schools were unable to read and write, whereas more than half of the mothers whose daughters were enrolled in private schools attended postsecondary school (Table 1).

### 3.2. Adolescents' Knowledge on Human Papillomavirus and Its Vaccination

Nearly two-thirds (63.4%) of students in public primary schools and three-fourths (73.4%) of students in private schools had some form of cervical cancer information, and there was a significant difference between schools in terms of level of acquiring cervical cancer information. In terms of obtaining HPV information, there is no statistical difference between public and private school students, even though a higher proportion of public students had received HPV information than the private students. Similarly, a lower proportion of students in private schools were aware of human papillomavirus vaccination when compared to students in public schools and the fact that this difference was statistically significant. The understanding of primary school students about the cause of cervical cancer did not show variation statistically between public and private schools (*X*^2^ = 0.394, *P* value = 0.295). However, the overall knowledge on HPV among primary school students showed a statistically significant difference by school ownership (*X*^2^ = 7.015, *P* value = 0.01) (Table 2).

### 3.3. HPV Vaccination and Healthcare Access–Related Characteristics

The proportion of adolescent students who had ever visited youth sexual and reproductive health services centers was 16.6% in public primary schools and 6.6% in privately owned schools, with no statistically significant difference by primary school ownership. Although the difference was not statistically significant, more public school students visited a health facility for sexual and reproductive health services during working hours than students from privately owned schools. The hours-of-service provision for youth reproductive health services was significantly lower for students enrolled in privately owned schools when compared to public students, and this difference was unlikely to be statistically significant. Furthermore, a higher proportion of private school students had to wait for reproductive healthcare services longer than public school students. Long waiting times, on the other hand, did not show a statistically significant difference in primary schools. In contrast to the preceding findings, service providers are more judgmental and unfriendly to students from private primary schools, and this difference was statistically significant (Table 3).

### 3.4. Health Belief Model Constructs and their Relationship with Willingness to Uptake Human Papillomavirus Vaccination

Health belief model was applied to select the best match constructs for the willingness to uptake human papillomavirus vaccination. Adolescent girls in the private primary schools demonstrated better scores of the HBM constructs (*P* < 0.001) compared with students in the public group. In all the constructs of the HBM, those students from the private schools had a strong and greater mean score than in public schools (*P* < 0.001). Thus, if we can apply the HBM of behavioral intervention to scale up the vaccination utilization, greater behavioral change and uptake would be resulted in private schools as compared to public school adolescents. All HBM constructs also showed a significant positive association with willingness to uptake HPV vaccination (*P* < 0.001) (Table 4).

### 3.5. Willingness to Uptake Human Papillomavirus Vaccination

Among primary school adolescents, the overall willingness to uptake the human papillomavirus vaccine was 50.6% (95% CI: 47.4-54). Adolescent girls attending public schools (61% (95% CI: 56.3-65.4)) were more likely to uptake HPV vaccination services than students attending private schools (40.2% (95% CI: 35.6-44.9) (*X*^2^ = −35.29, *P* value <0.001) (Figure 1).

### 3.6. Factors Associated with Willingness to Uptake Human Papillomavirus Vaccination

The bivariable logistic regression revealed that age group, school ownership type, grade level, maternal education, perceived susceptibility, perceived severity, perceived benefit, perceived barrier, cues to action, and self-efficacy all had a significant association with willingness to uptake HPV vaccination. Age group and maternal education status (illiterate, primary, and secondary) were not found to be significant in the multivariable logistic regression. School ownership type, maternal education (postsecondary), perceived barriers, cues to action, and self-efficacy were all predictors of willingness to uptake HPV vaccinations. Adolescents who attended public-owned primary schools were 1.9 times more likely to be willing to uptake human papilloma vaccine (AOR = 1.91; 95% CI: 1.4, 2.6) than adolescent students who attended privately owned schools. Adolescents from postsecondary school–educated mothers were twice as likely as illiterate mothers to uptake the human papillomavirus vaccine (AOR = 2.0; 95% CI: 1.3, 3.1). Adolescents with high cues to action were 1.9 times more likely than their counterparts to be willing to uptake the human papillomavirus vaccine (AOR = 1.9; 95% CI: 1.2, 3.1). Adolescent girls with high levels of self-efficacy were twice as likely as those with low levels of self-efficacy to be willing to take the human papillomavirus virus vaccine (AOR = 2.34; 95% CI: 1.2, 3.1). Adolescent students who perceived barriers as high were 55% less likely to accept HPV vaccination (AOR = 0.45, 95% CI: 0.31-0.66) than their counterparts (Table 5).

## 4. Discussion

This study aimed at comparing the differences in willingness to uptake HPV vaccine between students enrolled in public and privately owned primary schools and identified factors for willingness to uptake HPV vaccine. In this study, the overall willingness to uptake HPV vaccine was 50.6% (95% CI: 47.4, 54) among adolescent girls aged 10 to 19 years, and the *X*^2^ test revealed a significant difference between public-run and privately owned primary schools in terms of willingness to uptake the HPV vaccine (*P* value < 0.001). Only 61% (95% CI: 56.3, 65.4) of public-run primary schools and 40.2% (95% CI: 35.6, 44.9) of privately owned schools accepted to uptake human papillomavirus vaccine. As far as we are aware, this is the first study of its kind to compare willingness to uptake HPV vaccination in adolescent students of public versus private schools in Bahir Dar, Northwest Ethiopia, and this will be an impute for policy circle in maternal and reproductive health. In comparison to the general population, adolescent girls' resistance to HPV vaccination has increased rapidly, as suggested by previous studies. Several factors influenced the rapid emergence of HPV vaccine hesitancy, including parents' concerns that the vaccine will encourage risky adolescent sexual behavior, misinformation about the vaccine's efficacy and safety, and long- and short-term side effects [4, 26–28]. The study of the barriers to HPV vaccination uptake among adolescent female students, where there was a low rate of timely HPV vaccine use, was an important tool in reducing the health effects of the human papillomavirus. The average age of adolescent female students enrolled in both public and privately owned schools was 13.78 years and 13.74 years, respectively; however, there was a statistically significant difference in age groups between public and private primary school students.

According to the previous literature, HPV vaccination is recommended for prepuberty adolescent girls between the ages of 9 and 14 [14], provided that the majority of school students included in this study were found to be in the age groups targeted by WHO, and increasing HPV vaccination utilization among these population is mandatory. Hence, designing and facilitating healthcare service educations and other promotional strategy in accordance with the context demands should be implemented in Bahir Dar City in particular. However, in many resource-constrained countries, lack of access to healthcare education among females is an impediment that makes it more difficult to promote adolescent health, particularly in increasing willingness to uptake HPV vaccine. The study also discovered that maternal education was a predictor of willingness to uptake HPV vaccination as clearly identified in the multivariable regression modeling, similar to previous studies [22–24, 29, 30]. As a result, increasing formal education is beneficial for changing behavior to prevent and control cervical cancer, especially among the parents of the target population that is school adolescents. In the culturally sensitive societies like Ethiopia, mothers are the consultant and caretaker of their daughters such that if women are educated, it is believed that families are saved from any literacy-associated catastrophe.

Furthermore, in public schools, the level of knowledge regarding HPV vaccination and cervical cancer independently predicted the use of HPV vaccinations [22, 30–32], whereas in private elementary schools, there was no association between willingness to uptake HPV vaccination and level of knowledge about HPV vaccinations (*P* > 0.05). This was also supported by the findings of the *X*^2^ test, which revealed a significant difference in knowledge levels between public and private adolescent female students (*P* < 0.05). Existing studies also indicated that women who were educated about cervical cancer had a higher likelihood of knowledge and were more motivated to uptake the HPV vaccine [24].

The population found in this study was made up of adolescent female students, who are thought to be linked to the HPV vaccine hesitancy; however, if the vaccine coverage has targeted them in younger ages, it is one of the potential mechanisms used to reduce the disease infection rates. As a result, regardless of their knowledge characteristics, most healthcare professionals would prefer to advise adolescents on how to receive the vaccination at the prepubertal age rather than in the general population assuming that policymakers should be most concerned about the type of population being targeted and the role of healthcare providers in HPV vaccination supplementation program, given that these contexts are the most likely causes of any disparities between service provision and uptake. Participants in North Gondar [23], Debre Tabor [22], Debre Markos [29], and Bench Sheko zone [24], for example, were parents of school-aged children, whereas those in Jimma [30] were female high school students where HPV vaccine acceptance was highly reflected preadolescents.

High cues to action increased the likelihood of willingness to receive human papillomavirus vaccination. The current study discovered that adolescent girls with high cues to action were more likely to be willing to receive HPV vaccination services, correlating with the findings of other studies conducted in North Gondar, Ethiopia [33], Ghana [34], South Africa [35], Northern Cyprus [36], and the United States [37]. This can be explained by the fact that people with high cues to action on health-related behaviors are more likely to be persuaded by any available health information about HPV vaccine. Adolescents' cues to use the HPV vaccine to prevent cervical cancer may come from themselves or from relevant others. As a result, self-encouragement could take the form of a desire to use the HPV vaccine in anticipation of cervical cancer, whereas outside encouragement could come from family, a friend's invitation, and counseling from health professionals. Thus, program owners should consider either self-perception or the role of relevant others in promoting healthy behavioral change.

For Ethiopia, WHO recommended primary school–aged girls to be the primary target populations for HPV vaccination. Despite this recommendation, it is difficult to maintain high HPV vaccine uptake among eligible adolescents. Women who perceived a significant barrier to performing the behavior, for example, were less likely to perform the IVA test [38]. Because of poor health-seeking behavior and perceived barriers, the current study found that misunderstandings and misperceptions about the cause and prevention of cervical cancer were common. This study, as in the previous studies [39, 40], noted that a high perceived barrier reduced the likelihood of willingness to receive human papillomavirus vaccination. In other words, taking action to prevent a disease or seek treatment was influenced by perceived barriers, which were the barriers that arose when performing an action. This is because the experience of a person in determining health actions or utilizing health services was dominated by personal constraints. Accordingly, perceived barriers were a predictor of behavioral changes. As a result, before the nationwide expansion of cervical cancer prevention programs, it is critical to assess barriers to HPV vaccination acceptance and use through appropriate community-level studies [22, 29, 30]. Every country must take steps to understand the extent and nature of hesitancy at the community level on an ongoing basis and as a result, should develop a strategy to increase acceptance and demand for vaccination [28].

Attending school increases the likelihood of being willing to receive human papillomavirus vaccination. The willingness to receive human papillomavirus vaccination was 1.9 times higher among school girls. This finding is consistent with the studies from Ethiopia [33], South Africa [26, 35], and China [4]. The most likely explanation for this relationship is that HPV vaccination is the responsibility of the ministry of health, one of the public implementing agencies, which prioritizes public schools over private schools due to resource constraints, and that most private schools in Ethiopia are business-oriented and the fact that much promotional and health literacy activity may take place in public schools. Thus, it is suggested that adolescent girls should be vaccinated against HPV through conducting school-based health education promotional strategy, which was particularly effective in raising awareness and favorable attitudes toward HPV and should have influenced the acceptance of the vaccine. It is also commendable that incorporating HPV health education into existing school-based sexual health curricula would encourage HPV vaccination and increase its coverage.

Even though socioeconomic factors such as income status, family size, purchasing habits, and motivational factors were not investigated as potential determinants for HPV vaccination use, the current study found that adolescent girls with a high level of self-efficacy toward HPV vaccination were significantly associated with the willingness to accept HPV vaccination. This finding is consistent with the studies conducted in the world [41, 42]. It is plausible that HPV vaccine supplementation has to be targeted for task shifting in the grassroot community level of healthcare and adolescent girls in Ethiopia that tend to follow the advice and views of healthcare workers and community health workers. The recommendations may increase acceptance of vaccination against HPV among school adolescent girls. Furthermore, HPV vaccination decisions for adolescents, which are frequently parallel decisions, are a major motivator for vaccination [43].

Although efforts are exerted to reduce the limitation, this study would be susceptible to recall and social desirability biases. The study was also carried out during the period of the COVID-19 pandemic which had the potential to compromise the quality of the study results.

## 5. Conclusion

Adolescent girls in public primary schools were more likely to uptake HPV vaccination than those in private schools. Willingness to uptake HPV vaccination was found to be low as compared to the WHO target for resource-limited countries such as Ethiopia and was influenced by maternal education status, perceived barriers, cues to action, and self-efficacy in spite of healthcare access-related, income status, and socioeconomic factors becoming less important. As a result, greater emphasis should be placed on implementing a school-based educational program using a health belief model in the prevention and control of cervical cancer. To raise awareness, maternal education on cervical cancer and its prevention is also emphasized. Furthermore, appropriate weight should be given to the role of relevant others in raising HPV vaccination awareness through mass media and other channels to increase HPV vaccination utilization.

## Figures and Tables

**Figure 1:** Willingness to uptake human papillomavirus vaccination among public and private primary schools' adolescents in Bahir Dar City, Ethiopia (*n* = 820).

**Table 1:** Sociodemographic characteristics of public and private primary school adolescent girls in Bahir Dar City administration, 2021 (*n* = 820).

Variables	Public (**n** = 410)	Private (**n** = 410)	**X** ^2^	**P** value
	**n** (%)	**n** (%)		
Age mean (±SD)	13.86 (±1.76)	13.76 (±1.75)	13.745	0.013
Age group (year)				
10-14 yrs	251 (61.2)	318 (77.6)	3.037	0.008
15-19 yrs	159 (38.8)	92 (22.2)		
School grade level				
5-6 grades	121 (29.5)	182 (44.4)	0.885	0.35
7-8 grades	289 (70.5)	228 (55.6)		
Religion				
Orthodox	366 (89.3)	312 (76.1)	2.456	0.48
Muslim	39 (9.5)	64 (15.6)		
Others	5 (0.9)	34 (8.3)		
Family marital status				
Single	45 (11)	25 (6.1)	2.263	0.52
Married	301 (73.4)	347 (84.6)		
Widowed	31 (7.6)	14 (3.4)		
Divorced	33 (8.0)	24 (5.9)		
Mothers' education level				
Unable to read and write	199 (48.5)	14 (3.4)	3.553	0.470
Primary school	113 (27.6)	71 (17.3)		
Secondary school	53 (12.9)	101 (24.6)		
Postsecondary	45 (11)	224 (54.7)		
Mothers' employment status				
Yes	97 (23.7)	157 (38.3)	0.365	0.5
No	313 (76.3)	253 (61.7)		

**Table 2:** Knowledge on human papillomavirus among public and private primary school adolescent students in Bahir Dar City, Ethiopia, 2021 (*n* = 820).

Variables	Government (**n** = 410)	Private (*n* = 410)	*X* ^2^	*P* value
Ever heard/any information about cervical cancer				
Yes	260 (63.4)	301 (73.4)	6.146	0.008
No	150 (36.6)	109 (26.6)		
Ever heard/any information about HPV				
Yes	190 (46.3)	73 (17.8)	3.499	0.061
No	220 (53.7)	337 (82.2)		
Cervical cancer is caused by HPV				
Yes	93 (23.7)	60 (14.6)	0.394	0.295
No	317 (77.3)	350 (85.4)		
Ever heard/any information about the HPV vaccine				
Yes	128 (31.2)	62 (15.1)	7.015	0.01
No	282 (68.8)	348 (84.9)		
HPV knowledge (overall)				
Poor knowledge	154 (37.4)	120 (29.7)	6.336	0.007
Good knowledge	256 (62.4)	290 (70.3)		

**Table 3:** HPV vaccination and related healthcare access characteristics among public and private primary school students in Bahir Dar, Northwest Ethiopia, 2021 (*n* = 820).

Variables	Public	Private	*X* ^2^	*P* value
	*n* (%)	*n* (%)		
Adolescents have ever attended facilities for youth sexual and reproductive health service (SRH) (*n* = 820)				
Yes	68 (16.6)	27 (6.6)	0.769	0.222
No	342 (83.4)	383 (93.4)		
Period of adolescents' most recent visit to a health facility for SRH services (*n* = 95)				
Working hours	48 (70.9)	17 (66)	0.908	0.635
Out of working hours	20 (29.1)	10 (34)		
Youth reproductive health service hours are inconvenient (*n* = 95)				
Yes	37 (54.4)	19 (70.3)	0.979	0.573
No	31 (45.6)	8 (29.6		
Fear of being seen by parents or others when you visit RH service (*n* = 95)				
Yes	39 (57.4)	19 (70.3)	0.133	0.8
No	29 (42.6)	8 (29.6)		
Reproductive health service waiting hours are too long (*n* = 95)				
Yes	41 (60.3)	19 (70.3)	0.583	0.291
No	27 (39.7)	8 (29.6)		
Service providers are judgmental and unfriendly (*n* = 95)				
Yes	29 (42.6)	19 (70.3)	3.033	0.041
No	39 (57.4)	8 (29.6)		
Feel embarrassment at seeking RH services (*n* = 95)				
Yes	23 (33.8)	13 (48.1)	1.286	0.178
No	45 (67.2)	14 (51.9)		

**Table 4:** Health belief model constructs on willingness to uptake HPV vaccination among primary school adolescent girls in Bahir Dar City administration, Ethiopia, 2021 (*n* = 820).

Health belief model constructs on willingness to uptake HPV vaccination	Loading factor	Public (**n** = 410)		Private (**n** = 410)		**X** ^2^	**P** value
		Mean	Standard deviation	Mean	Standard deviation		
Perceived susceptibility	0.44	12.40	(5.18)	12.82	(±4.81)	30.06	0.018
Perceived severity	0.73	14.24	(4.60)	17.03	(±3.67)	130.01	<0.001
Perceived benefit		13.31	(3.60)	20.79	(±2.08)	20	<0.001
Perceived barrier	0.53	14.05	(4.44)	14.98	(±4.16)	40	<0.001
Cue to action	0.8	13.73	(4.80)	16.28	(±4.51)	35	<0.001
Self-efficacy	0.76	14.24	(4.60)	17.03	(±3.67)	44	<0.001

**Table 5:** Factors associated with the willingness to uptake HPV vaccination among primary school students in Bahir Dar City, Ethiopia (*n* = 820).

Variables	Willingness to uptake HPV vaccination		COR (95% CI)	AOR (95% CI)
	Yes (**n**, %)	No (**n**,%)		
School ownership (type)				
Public	250 (61)	160 (39)	2.32 (1.75, 3.0)	1.91 (1.4, 2.6)
Private	165 (40.2)	245 (59.8)	1	1
Age groups				
10-14 yrs	302 (53.1)	267 (46.9)	1	1
15-19 yrs	103 (41)	148 (59)	1.62 (1.2, 2.19)	1.1 (0.77, 1.56)
Adolescent grade level				
5-6 grades	173 (57.1)	130 (42.9)	1	1
7-8 grades	232 (44.9)	285 (55.1)	1.63 (1.22, 2.17)	1.53 (0.13, 2.18)
Mother education				
Illiterate	125 (58.7)	88 (41.3)	1	1
Primary	92 (50)	92 (50)	1.38 (0.91, 2.07)	1.2 (0.78, 1.85)
Secondary	78 (50.6)	76 (49.4)	1.41 (0.92, 2.16)	1.38 (0.87, 2.17)
Postsecondary	120 (44.6)	149 (53.4)	1.76 (1.31, 2.90)	2.0 (1.29, 3.05)
Perceived barrier				
High	282 (68)	310 (76.5)	0.65 (0.47, 0.88)	0.45 (0.31, 0.66)
Low	133 (32)	95 (23.5)	1	1
Cue to action				
High	376 (90.6)	322 (79.5)	2.48 (1.72, 3.70)	1.92 (1.20, 3.07)
Low	39 (9.4)	83 (20.5)	1	1
Perceived susceptibility				
Low	26 (6.3)	53 (13.1)	1	1
High	389 (93.7)	352 (86.9)	2.3 (1.37, 3.68)	1.4 (0.79, 2.48)
Perceived benefit				
Low	8 (1.9)	28 (6.9)	1	1
High	407 (98.1)	377 (93.1)	3.35 (1.56, 7.19)	1.25 (0.50,3.10)
Self-efficacy				
High	361 (87)	284 (70.1)	2.84 (1.99,4.06)	2.34 (1.58,3.48)
Low	54 (13)	121 (29.9)	1	

## Data Availability

All relevant materials and data supporting the findings of this study are freely available. All relevant data are within the manuscript and its Supporting Information files. When necessary, please contact destad2a@gmail.com.

## Abbreviations

CI: Confidence interval
AOR: Adjusted odds ratio
HPV: Human papillomavirus
SSA: Sub-Saharan Africa
HBM: Health belief model
MPH/RH: Master of health in reproductive health
IRB: Institute review board.
